# Food deserts exposure, density of fast-food restaurants, and park access: Exploring the association of food and recreation environments with obesity and diabetes using global and local regression models

**DOI:** 10.1371/journal.pone.0301121

**Published:** 2024-04-18

**Authors:** Jae In Oh, KangJae Jerry Lee, Aaron Hipp

**Affiliations:** 1 Department of Parks, Recreation & Tourism Management, North Carolina State University, Raleigh, North Carolina, United States of America; 2 Department of Parks, Recreation & Tourism, University of Utah, Salt Lake City, Utah, United States of America; 3 Center for Geospatial Analytics, North Carolina State University, Raleigh, North Carolina, United States of America; Villanova University, UNITED STATES

## Abstract

To prevent obesity and diabetes environmental interventions such as eliminating food deserts, restricting proliferation of food swamps, and improving park access are essential. In the United States, however, studies that examine the food and park access relationship with obesity and diabetes using both global and local regression are lacking. To guide county, state, and federal policy in combating obesity and diabetes, there is a need for cross-scale analyses to identify that relationship at national and local levels. This study applied spatial regression and geographically weighted regression to the 3,108 counties in the contiguous United States. Global regression show food deserts exposure and density of fast-food restaurants have non-significant association with obesity and diabetes while park access has a significant inverse association with both diseases. Geographically weighted regression that takes into account spatial heterogeneity shows that, among southern states that show high prevalence of obesity and diabetes, Alabama and Mississippi stand out as having opportunity to improve park access. Results suggest food deserts exposure are positively associated with obesity and diabetes in counties close to Alabama, Georgia, and Tennessee while density of fast-food restaurants show positive association with two diseases in counties of western New York and northwestern Pennsylvania. These findings will help policymakers and public health agencies in determining which geographic areas need to be prioritized when implementing public interventions such as promoting healthy food access, limiting unhealthy food options, and increasing park access.

## 1. Introduction

Obesity and diabetes are health outcomes associated with premature death in the U.S. [1, 2]. The obesity rate among adults reached 41.9% in 2017-March 2020 and diabetes reached 11.3% in 2019 [3, 4]. Today, the medical expenditure for treating each disease costs more than $300 billion annually [3, 5], and the expenditure is likely to rise as both diseases are expected to increase continuously over the next decades [6, 7]. Furthermore, obesity and diabetes rates are disproportionately higher among racial and ethnic minorities and people with low socioeconomic status (SES), raising a serious health inequity issue [8–10].

To cope with the increasing rate of obesity and diabetes, as well as their disproportionate impact on non-White communities and low SES groups, many studies have investigated causes of these diseases and potential solutions. They have identified that excessive energy intake and insufficient physical activity are two main culprits [11–13]. Consequently, researchers have explored different strategies to prevent these two diseases and found that individual-level preventive approaches such as encouraging a healthy diet and regular exercise yield meaningful results [14–16].

A recent comprehensive review has demonstrated an association between active engagement in physical activities and a reduced risk of developing obesity, diabetes, and coronary heart disease [17]. However, an association was not found between physical activity and hypertension. This suggests that physical activity may have a more significant health-protective impact on obesity and diabetes compared to hypertension, another prominent factor contributing to premature death [18]. Also, according to a perspective paper, about 90% of type 2 diabetes is attributable to an excess of body weight [19] and increase in obesity is associated with the rise of diabetes [20]. Therefore, addressing each health issue, either obesity or diabetes, may not be feasible without simultaneously addressing the other issue.

A growing body of research found certain built environment characteristics promote or hinder healthy diet and physical activity. Cross-sectional studies confirmed that the availability of supermarkets and the density of fast-food restaurants were positively associated with a healthy and low-quality diet, respectively [21–23]. Similarly, the availability of recreation resources (i.e., parks and trails) was positively associated with the frequency of physical activity [24].

In the U.S., unhealthy food environments, such as the presence of food deserts and high density of fast-food restaurants, are considered as contributing factors to the increasing rates of obesity and diabetes rates [25, 26]. Existing literature define residential areas located far from large food retailers and do not have easy access to transportation as ‘food deserts’ and areas inundated with fast-food restaurants that sell unhealthy energy-dense foods and beverages as ‘food swamps’ [27, 28]. Previous study found that food swamps have more close association with obesity than food deserts among U.S adults [29].

Despite the significant relationships between food environment (FE), park access (PA), diet, and physical activity, most national-level studies in the U.S. do not incorporate both FE and PA simultaneously in their analyses to identify their impact on obesity and diabetes [30–32]. These studies focused on the association of recreation resources with either obesity or diabetes but left out FE indicators in their analyses [31, 32] or examined solely the relationship between FE and diabetes [28, 30]. Therefore, by incorporating both FE and PA measures, we can gain a more holistic understanding of the relationship between environmental factors and these two chronic diseases.

Today, the degree to which FE and PA measures are associated with these two diseases at the local level based on geographically weighted regression has remained largely understudied. Therefore, we have limited understanding of the association between FE and PA measures and geographic clusters of obesity and diabetes. Spatial clusters of obesity and diabetes in the southeastern U.S., a region where people tend to have lower income than other regions, have been consistently found in previous studies [9, 31, 33, 34]. While a recent study confirmed that neighborhoods in the southern U.S lack both food and physical activity resources [35], we have limited evidence that confirms whether obesity and diabetes are strongly associated with FE or PA measures, and which states in southern U.S show strong or weak association with those measures.

Several studies examined the relationships between access to food and parks and their impact on physical activity, obesity, or diabetes through geographically weighted regression [31, 36–39]. While these studies also used FE and PA measures, variations exist in the unit of analysis, data included in the research, and the methodologies used to assess park and food environment. For example, one study used measures of exercise opportunities encompassing commercial recreational facilities and parks [37], while another study focused exclusively on tree canopy coverage [36]. One study used network-based park accessibility but did not adjust for food environment in their analysis on obesity prevalence [31]. Although studies that focused on similar research topics and used same regression models exist, we assume direction and degree of relationship between park, food environment, obesity, and diabetes may vary depending on the choice of different accessibility measures and whether both park and food environment are included in the analysis or not.

This study aims to answer to what degree obesity and diabetes belt observed in the southern U.S is attributable to the lack of healthy grocery stores (i.e., food deserts exposure), density of fast-food restaurants, and limited park access measured based on network distance. Specifically, this study seeks to address four research questions: 1) In which regions of the U.S do FE (i.e., food deserts exposure and density of fast-food restaurants) and PA spatially correlate with obesity and diabetes? (2) To what degree are FE and PA associated with obesity and diabetes in a global regression model (i.e., nationally)? (3) What is the spatial heterogeneity of FE and PA with obesity and diabetes? (4) To what extent are the environmental characteristics associated with obesity and diabetes clusters previously identified in the southern United States. We hypothesize that A) food deserts exposure and density of fast-food restaurants will show positive relationship with obesity in both global and local levels; B) food deserts exposure and density of fast-food restaurants will show positive relationship with diabetes in both global and local levels; C) park access will show inverse relationship with obesity in both global and local levels; and D) park access will show inverse relationship with diabetes in both global and local levels.

## 2. Methods

### 2.1 Data

This study used a secondary dataset from the 2019 County Health Rankings (CHR), a health measurement program affiliated with Robert Wood Johnson Foundation and the University of Wisconsin Population Health Institute, to obtain information about adult obesity, diabetes, gender, income, race, and unemployment in the 3,108 counties of the contiguous U.S. Information on grocery store access and fast-food restaurant density were based on the Food Environment Atlas from the U.S. Department of Agriculture (USDA). Data from the Food Environment Atlas are publicly available at the census tract, county, and state level across the U.S., and it is updated regularly. We used the March 2018 county-level data to best match CHR data.

2018 ParkServe data from the Trust for Public Land was used as the measure of park access. The agency operationalized the 10-minute walkable service area of parks across the U.S. This information was developed by taking into account real-world street networks using Geographic Information Systems (GIS). To extract accessible parks within each county in the contiguous U.S., we performed the spatial analysis by using the dissolve tool, multipart to single part tool, and intersect tool from ArcGIS version 10.6 software.

#### 2.1.1 Outcome variables

Obesity and diabetes rates of individual counties were the outcome variables of this study. CHR obesity rate was measured based on the body mass index (BMI) of individuals who participated in the Centers for Disease Control and Prevention (CDC)’s Behavioral Risk Factor Surveillance Survey and were aggregated to county level. Specifically, the CDC developed the obesity rate of each county by extracting the percentage of the adults aged over 20 who reported a BMI greater than or equal to 30 kg/m^2^. CHR diabetes rate was also from Behavioral Risk Factor Surveillance Survey, which calculated the percentage of adults over 20 years old who answered “yes” to the question, “Has a doctor ever told you that you have diabetes?”.

#### 2.1.2 Independent variables

Food environment (FE) and park access (PA) in each county were used as independent variables. FE was operationalized using two variables retrieved from Food Environment Atlas, the online mapping tool launched by USDA [40] U.S. Department of Agriculture, Economic Research Service. USDA [40] provide FE data such as the percentage of people who have low access to grocery stores (i.e. food deserts exposure) and the density of fast-food restaurants. It was considered low access if a supermarket, supercenter, or large grocery store was located more than 1 mile (if in urban area) or more than 10 miles (if in a rural area) from the center of the 0.5 kilometer-square grid cells assigned across each county.

According to USDA [41], 1-mile and 10-mile cutoffs were selected based on the statistical data. For example, in urban areas, 29% of individuals with low incomes residing in low-income areas were situated within a half-mile radius of a supermarket, while an additional 42% fell within the distance range between half a mile and one mile. In rural areas, most people living outside walking distance to a store and do not have a vehicle in rural areas lived between 1 mile and 10 miles from a supermarket.

In U.S., supermarkets have long been used as a proxy for healthy food stores, as they have been found to offer a greater selection of healthy foods compared to small family-owned businesses (mom-and-pop stores) and convenience stores [42]. Healthy foods include fruits and vegetables, and previous studies have shown that proximity to supermarkets and grocery stores is associated with a higher intake of fruits and vegetables [43, 44].

According to USDA [40], the process to measure access to grocery stores is as follows; block-level population data from the American Community Survey was allocated down to the grid (0.5-kilometer square grid) cells and then the population within grid cells who have low access to grocery stores was counted accordingly. The number of people in each grid cell living more than 1 mile or 10 miles from the supermarket in urban or rural areas respectively was aggregated to the county level. This aggregated population data were divided by the total population within the county to calculate the percentage of people who have low access to grocery stores at the county level.

The density of fast-food restaurants (FFR) was estimated based on the number of FFR per 1,000 county residents. USDA referred to limited-service restaurants, classified in North American Industry Classification System (NAICS) code 722511, as FFR. Stores primarily engaged in providing food services where patrons generally order or select items and pay before eating are included in the limited-service restaurants category [40].

As a measure of PA, we used service areas within a 10-minute walk from a park across the U.S and this data was originally from The Trust for Public Land’s ParkServe database. The Trust for Public Land used Esri’s Street Map Premium network dataset to consider physical barriers that can influence physical accessibility. These barriers include highways, train tracks, and rivers not connected to bridges [45]. We employed this network-based accessibility measure, as recommended by a systematic literature review [46], to confirm greenness access. Measure reflects the accessibility of parks and green spaces by walking not impeded by barriers mentioned above.

#### 2.1.3 Covariates

We included age, car ownership, education, gender, income, race, and unemployment as covariates because demographic and socio-economic factors were frequently associated with obesity and diabetes from previous studies [47, 48]. Table 1 summarizes all the study variables and related data sources.

**Table 1:** Description of variables.

Variables	Description	Data Source
Percent Obesity	Percentage of the adult population (age 20 and older) that reports a body mass index (BMI) greater than or equal to 30 kg/m2	CHR
Percent Diabetes	Percentage of adults aged 20 and above with diagnosed diabetes	CHR
Percent White	Percentage of Non-Hispanic White	CHR
Percent Black	Percentage of Non-Hispanic Black	CHR
Percent Hispanic	Percentage of Hispanic	CHR
Percent Female	Percentage of population that is female	CHR
Percent unemployed	Percentage of population aged 16 and older that is unemployed but seeking work	CHR
Percent bachelor’s	Percent of adults with a bachelor’s degree or higher	CHR
degree or higher		
Median household	Median income where half of households in a county earn more and half of households earn less	CHR
income ($)		
Median age	Median age of the total population in a single county	ACS
Percent households	Percentage of households that own a car	ACS
that own a car		
Percent accessible	Percentage of the publicly accessible parks within 10-minute walk	TPL
park areas		
Percent of people	Percentage of people in a county living more than 1 mile from a supermarket, supercenter, or large grocery store if in an urban area, or more than 10 miles from a supermarket or large grocery store if in a rural area.	FEA
living in food desert		
area		
Density of fast-food	Number of fast-food restaurants / 1,000 population	FEA
restaurants		

Note: CHR represents County Health Rankings (accessed from https://www.countyhealthrankings.org/explore-health-rankings/rankings-data-documentation/national-data-documentation-2010-2019); ACS represents the American Community Survey; TPL represents Trust for Public Land;

FEA represents Food Environment Atlas (accessed from https://www.ers.usda.gov/data-products/food-access-research-atlas/download-the-data/#Current%20Version)

### 2.2 Statistical analysis and Local Indicators of Spatial Association (LISA)

#### 2.2.1 Global and local spatial autocorrelation

Observations from the specific geographic unit are likely to be affected by nearby spatial units, resulting in the issue of spatial autocorrelation [49]. Global Moran’s I statistic helps determine the presence of spatial autocorrelation from the variable of interest across the entire study area and uncovers the overall tendency of spatial concentration [50]. We computed Global Moran’s I statistic by using the GeoDa software [51] and confirmed the presence of positive spatial autocorrelation from both obesity and diabetes rates (specific measures are described in the Results section).

We also used Local Moran’s I statistic to examine the extent of spatial effects and to identify statistically significant clusters of spatial autocorrelation [52]. Although Global Moran’s I helps confirm the overall degree of spatial autocorrelation, it cannot specify areas where similar values are spatially clustered [53]. Conversely, Local Moran’s I can identify the degree of spatial autocorrelation in neighborhood levels and locate areas where significant spatial autocorrelation is present.

In this study, we used Bivariate Local Indicators of Spatial Autocorrelation (BiLISA) to identify spatial clusters where a single variable (e.g., FE or PA) in a spatial unit strongly correlates with another variable (e.g., obesity or diabetes) in neighboring spatial units [54]. Clusters from BiLISA consist of four clusters, namely High-High (HH), High-Low (HL), Low-High (LH), and Low-Low (LL) clusters and these clusters are generated based on the value of Local Moran’s I. We created these clusters based on the default setting of 9,999 permutations and a p-value of 0.05 from GeoDa software.

#### 2.2.2 Spatial regression models

This study used the spatial regression method, which addresses the issue of spatial dependency between each geographic unit [54] when exploring the global relationship between variables. The Lagrange Multiplier (LM) test available from GeoDa software helps to determine which spatial regression model is more appropriate for the analysis. There are two kinds of LM test: LM-Lag and LM-Error. Anselin [55] recommended using the one that rejects the null hypothesis, which proposes no spatial autocorrelation. When both tests reject the null hypothesis, the rule of thumb is to select the model with statistically significant Robust LM Diagnostics [55]. If both models present significant Robust LM Diagnostics, choosing the one that has larger values of the test statistic is recommended.

Table 2 presents the results of the Robust LM Diagnostics test for the two dependent variables, the obesity and diabetes rates. The results show the Robust LM values of Spatial Error Model (SEM) were higher than Spatial Lag Model (SLM) when both obesity and diabetes rates were used as dependent variables. Therefore, SEM was used as the final model.

**Table 2:** Results of Lagrange Multiplier test.

Variable	Test	Degree of Freedom	Value	*p*-value
Obesity	LM (SLM)	1	1943.285	0.000
	LM (SEM)	1	3392.661	0.000
	Robust LM (SLM)	1	81.934	0.000
	Robust LM (SEM)	1	1531.310	0.000
Diabetes	LM (SLM)	1	2491.256	0.000
	LM (SEM)	1	3831.273	0.000
	Robust LM (SLM)	1	348.020	0.000
	Robust LM (SEM)	1	1688.037	0.000

The equation for SEM is as follows:

Y=βX+λWε+ξ

where Y is the dependent variable; β is regression coefficient; X is the independent variable; λ is the spatial autocorrelation parameter; Wε is the spatial weight matrix; and ξ is the homoscedastic and independent error term.

#### 2.2.3 Geographically weighted regression

In addition to SEM, we performed geographically weighted regression (GWR) to explore the local spatial non-stationarity between FE and PA with obesity and diabetes at county levels. While the SEM helps identify the global relationship between variables, it does not account for the effects of spatial heterogeneity, and thus cannot explain the local relationship between variables. GWR can overcome this limitation as it measures localized parameter estimates and provides local variations in the association between independent and dependent variables. GWR determines the spatial scope of spatial dependency by setting the number of neighbors using kernel bandwidth [56] and calculates local regression coefficient by using a distance decay kernel function, which assigns more weight to the observations close to each other than observations located further away [57]. In this study, we used adaptive bi-square kernel bandwidth to account for different spatial extent or size of counties, and optimal bandwidth (number of neighbors) was selected based on golden bandwidth selection method.

The equation for GWR model can be expressed as follows:

$$yi=\beta_{0}(ui,vi)+\underset{\text{k}}{\sum }\beta_{k}\left(u_{i},v_{i}\right){\text{x}}_{\text{ik}}+\varepsilon i$$

where *yi* is the dependent variable, *β*_0_(*ui*,*vi*) denotes intercept at location i, and *β*_*k*_(*u*_*i*_,*v*_*i*_) represents local regression coefficient at location i. x_ik_ is the kth independent variable at location i and *εi* denotes random error term at location i. GWR was performed in MGWR 2.2 [58] and to visualize spatial heterogeneity, local coefficients for each county were mapped by using sf [59], tigris [60], and tmap [61] packages from R Software version 4.1.1 [62].

## 3. Results

### 3.1 Descriptive statistics and correlation analysis

Descriptive statistics of the study variables are summarized in Table 3. 3,108 counties across the contiguous U.S. were included in statistical analyses. Bivariate correlations between study variables are summarized in Table 4. Statistically significant correlation coefficients ranged from 0.038 to 0.719, indicating the presence of moderate correlation between variables [63]. Specifically, education level (bachelor’s degree or higher) and income showed highest correlation (0.719) followed by obesity and diabetes (0.672), which indicates both diseases can occur at the same time. We decided to use each risk factor separately in distinct regression models as coefficients between obesity and diabetes may affect the goodness of fit in regression model. While education and income are highly correlated, we included both variables because a previous study found that the relationship between income and food purchasing behavior was only marginally affected after adjusting for education [64].

**Table 3:** Descriptive statistics (N = 3,108).

Variables	Mean	SD	Min	Max
Percent Obesity	32.081	4.583	13.600	49.500
Percent Diabetes	11.661	2.587	3.300	20.900
Percent White	76.632	19.811	2.760	97.923
Percent Black	9.047	14.366	0	85.330
Percent Hispanic	9.516	13.820	0.515	96.323
Percent Female	49.929	2.183	26.575	57.004
Percent unemployed	4.577	1.570	1.624	19.066
Percent bachelor’s degree or higher	21.191	9.294	5.000	78.000
Median household income ($)	50952.390	13424.140	22679.000	136,191.000
Median age	41.188	5.350	21.600	66.400
Percent households that own a car	93.550	3.670	22.137	100
Percent accessible park areas	4.558	9.669	0	95.774
Percent people living in food desert area	22.682	19.301	0	100
Density of fast-food restaurants	57.847	30.455	0	555.556

**Table 4:** Bivariate correlations between covariates (CV), independent variables (IV), and dependent variables (DV).

Variables	CV 1	CV 2	CV 3	CV 4	CV 5	CV 6	CV 7	CV 8	CV 9	IV 1	IV 2	IV 3	DV 1	DV 2
% Unemployment (CV 1)	1													
Median household income (CV 2)	-0.438*	1												
% Black (CV 3)	0.306*	-0.240*	1											
% Hispanic (CV 4)	0.075*	0.029	-0.109*	1										
% White (CV 5)	-0.311*	0.127*	-0.618*	-0.626*	1									
% Female (CV 6)	0.038	0.038	0.143*	-0.150*	-0.008	1								
Median age (CV 7)	0.013	-0.119*	-0.202*	-0.318*	0.460*	0.010	1							
% Bachelor’s degree or higher (CV 8)	-0.370*	0.719*	-0.088*	-0.005	0.011	0.183*	-0.171*	1						
% Vehicle ownership (CV 9)	-0.356*	0.280*	-0.434*	-0.013	0.361*	-0.146*	0.174*	0.077*	1					
% Accessible park areas (IV 1)	-0.014	0.337*	0.068*	0.047	-0.130*	0.138*	-0.122*	0.473*	-0.332*	1				
% People living in food desert area (IV 2)	-0.113*	0.007	-0.074*	0.108*	-0.063*	-0.106*	0.070*	0.057	0.166*	-0.080*	1			
Density of fast-food restaurants (IV 3)	-0.048	0.171*	0.048	0.075*	-0.092*	0.179*	-0.186*	0.332*	-0.116*	0.287*	-0.101*	1		
% Obesity (DV 1)	0.255*	-0.460*	0.323*	-0.292*	-0.018	0.084*	-0.062	-0.558*	-0.149*	-0.308*	-0.096*	-0.197*	1	
% Diabetes (DV 2)	0.429*	-0.563*	0.433*	-0.302*	-0.090*	0.196*	0.205*	-0.567*	-0.257*	-0.214*	-0.149*	-0.161*	0.672*	1

*p*-values in parentheses (note: p-value was adjusted based on Bonferroni correction. Alpha level (0.05) divided by number of tests (N = 91))

* p<0.0005

We further examined potential multicollinearity between covariates and independent variables by confirming variance inflation factor (VIF) from R software version 4.1.1 [62]. The mean VIF was 2.89 and VIF score ranged from 1.65 to 9.29, which indicates no signs of excessive multicollinearity [65].

### 3.2 Spatially correlated patterns of FE/PA with obesity/diabetes

We examined the spatial pattern of FE and PA with obesity and diabetes across the contiguous U.S. at the county level by using a BiLISA analysis.

#### 3.2.1 Food deserts exposure and obesity

As shown in Fig 1(A), the HH clusters of food deserts exposure and obesity were more prevalent in southern and Midwest states. LL clusters were concentrated around large cities in the western and northeastern U.S.

**Fig 1:** Bivariate LISA cluster map for limited grocery store access (GSA) and obesity rates. **(a).** Stamen map tiles (Map tiles by Stamen Design, under CC BY 4.0. Data by OpenStreetMap, under ODbL) were used to create the map. **(b). Bivariate LISA cluster map for fast-food restaurants (FFR) density and obesity rates.** Stamen map tiles (Map tiles by Stamen Design, under CC BY 4.0. Data by OpenStreetMap, under ODbL) were used to create the map. **(c). Bivariate LISA cluster map for limited grocery store access (GSA) and diabetes rates.** Stamen map tiles (Map tiles by Stamen Design, under CC BY 4.0. Data by OpenStreetMap, under ODbL) were used to create the map. **(d). Bivariate LISA cluster map for fast-food restaurants (FFR) density and diabetes rates.** Stamen map tiles (Map tiles by Stamen Design, under CC BY 4.0. Data by OpenStreetMap, under ODbL) were used to create the map. **(e). Bivariate LISA cluster map for park access and obesity rates.** Stamen map tiles (Map tiles by Stamen Design, under CC BY 4.0. Data by OpenStreetMap, under ODbL) were used to create the map. **(f). Bivariate LISA cluster map for park access and diabetes rates.** Stamen map tiles (Map tiles by Stamen Design, under CC BY 4.0. Data by OpenStreetMap, under ODbL) were used to create the map.

#### 3.2.2 Density of fast-food restaurants and obesity

Fig 1(B) shows clusters of fast-food restaurants (FFR) density and obesity rates. HH clusters describing areas with counties of high FFR density spatially correlating with counties with high obesity rates were situated in southern states, western states of the Midwest, and Appalachian states such as Kentucky, Ohio, South Carolina, and West Virginia, as well as Indiana. LL clusters were dispersed across Rocky Mountain states and Arizona.

#### 3.2.3 Food deserts exposure and diabetes

As described in Fig 1(C), regarding food deserts exposure and diabetes, the HH clusters were concentrated in the southern states such as Arkansas, Louisiana, Mississippi, and Oklahoma, and dispersed across additional states in the South. Like LL clusters in Fig 1(A), LL clusters were largely located at large cities in the western and northeastern U.S.

#### 3.2.4 Density of fast-food restaurants and diabetes

The bivariate LISA cluster map for FFR density and diabetes rates is shown in Fig 1(D). HH clusters depicting areas where counties with a high density of FFR surrounded by counties with high diabetes rates were in southern and Appalachian states. LL clusters were situated in areas near large cities in the Midwest, such as Minneapolis and St. Louis, as well as in the Rocky Mountain region, including Albuquerque and Denver.

#### 3.2.5 Park access and obesity

As shown in Fig 1(E), concerning park access and obesity rates, LH clusters, indicating areas where counties with low percentages of park areas within a 10-min walk (accessible park areas) spatially correlate with counties showing high obesity rates, were dispersed across states in the southern U.S such as Arkansas, Kentucky, Louisiana, and West Virginia. HH clusters had the smallest number of county clusters. LL clusters were in largely rural areas in Rocky Mountain states. HL clusters were largely found in California, Colorado, Massachusetts, and New York State where average salary tends to be higher than other states [66].

#### 3.2.6 Park access and diabetes

Fig 1(F) describes LISA cluster maps that show the spatially correlated patterns between park access and diabetes rates. LH clusters denoting areas where counties with low percentage of accessible park areas surrounded by counties with high diabetes rates were in a few regions in southern states that belong to Arkansas, Florida, Louisiana, and West Virginia. LL clusters were largely found in Rocky Mountain states and states in the Midwest. Like park access and obesity, HL clusters were identified in high income states such as California, Colorado, Massachusetts, and New York State.

### 3.3 Global regression results from spatial error model (SEM)

In this study, the Global Moran’s I value of obesity rate was 0.528 (*p* < 0.0001) and that of diabetes rate was 0.593 (*p* <0.0001), indicating the existence of positive spatial autocorrelation from the two dependent variables. Therefore, we performed spatial regression in addition to Ordinary Least Squares (OLS) regression. As SEM proves to be a better model than OLS regression, we only summarized the global regression results from SEM.

As shown in Model 2 from Table 5, PA (*B* = -0.033, *p* <0.001), proportion of Hispanics (*B* = -0.099, *p* <0.001), non-Hispanic Whites (*B* = -0.054, *p* <0.001), median age (*B* = -0.129, *p* <0.001), and education (*B* = -0.239, *p* <0.001) were negatively associated with obesity at the county level. On the other hand, proportion of non-Hispanic Blacks (*B* = 0.028, *p* <0.01), females (*B* = 0.169, *p* <0.001), unemployment (*B* = 0.175, *p* <0.001), and vehicle ownership (*B* = 0.067, *p* <0.001) were positively associated with obesity.

**Table 5:** Global regression results from OLS regression and SEM.

	Model 1: OLS Obesity	Model 2: SEM Obesity	Model 3: OLS Diabetes	Model 4: SEM Diabetes
Variables	Coeff.	Coeff.	Coeff.	Coeff.
	(S.E)	(S.E)	(S.E)	(S.E)
% Black	0.042***	0.028**	0.022***	-0.030***
	(0.009)	(0.010)	(0.004)	(0.005)
% Hispanic	-0.123***	-0.099***	-0.072***	-0.089***
	(0.009)	(0.010)	(0.005)	(0.005)
% White	-0.014	-0.054***	-0.036***	-0.071***
	(0.009)	(0.008)	(0.004)	(0.004)
Median age	-0.205***	-0.129***	0.070***	0.116***
	(0.013)	(0.012)	(0.006)	(0.006)
% Bachelor’s degree or higher	-0.271***	-0.239***	-0.121***	-0.094***
	(0.010)	(0.009)	(0.005)	(0.004)
% Female	0.275***	0.169***	0.228***	0.132***
	(0.028)	(0.023)	(0.014)	(0.011)
% Unemployed	0.038	0.175***	0.178***	0.102**
	(0.045)	(0.048)	(0.022)	(0.023)
Median household income ($)	-0.038×10^−4^	0.110×10^−4^	-0.229×10^-^***	-0.081×10^−4^*
	(0.068×10^−4^)	(0.071×10^−4^)	(0.034×10^−4^)	(0.033×10^−4^)
% Vehicle ownership	0.009	0.067***	0.005	-0.007
	(0.020)	(0.019)	(0.010)	(0.009)
% Accessible park areas	-0.036***	-0.033***	-0.001	-0.012***
	(0.008)	(0.007)	(0.004)	(0.003)
% People living in food desert area	0.583×10^−3^	-0.077×10^−3^	-0.009***	0.005×10^−1^
	(0.003)	(0.003)	(0.002)	(0.001)
Density of fast-food restaurants	-0.006**	-0.001	-0.588×10^−3^	-0.001
	(0.002)	(0.002)	(0.001)	(0.0008)
Intercept	34.150***	31.340***	3.297***	9.546***
	(2.475)	(2.197)	(1.231)	(1.038)
N	3108	3108	3108	3108
R-squared	0.523	0.701	0.629	0.793
AIC	16007.400	14762.600	11667.500	10081.300

*p*-values in parentheses.

* p<0.05,

** p<0.01,

*** p<0.001

In Model 4, PA (*B* = -0.012, *p* <0.001), proportion of non-Hispanic Blacks (*B* = -0.030, *p* <0.001), Hispanics (*B* = -0.089, *p* <0.001), non-Hispanic Whites (*B* = -0.071, *p* <0.001), education (*B* = -0.094, *p* <0.001), and median household income (*B* = -0.0000081, *p* <0.05) were negatively associated with diabetes. Proportion female (*B* = 0.132, *p* <0.001), median age (*B* = 0.116, *p* <0.001), and unemployment (*B* = 0.102, *p* <0.001) were positively associated with diabetes.

From both Model 2 and Model 4, PA showed an inverse relationship with obesity and diabetes. FE measures, however, did not show a statistically significant relationship with obesity and diabetes.

### 3.4 Local regression results from geographically weighted regression (GWR)

Local R-squared values of GWR when obesity was set as the dependent variable are displayed in Fig 2. As illustrated from Fig 2, the GWR model showed high performance (R-squared at a range of 0.666–0.816) in Rocky Mountain states, northeastern states, and southern states including Alabama, Florida, Mississippi, North Carolina, and South Carolina. Areas where the explanatory power of the GWR model is relatively small (R-squared at a range of 0.226–0.409) were found in Midwest regions and several southern states such as Georgia, Kentucky, Tennessee, and Texas.

**Fig 2:** Local R-squared estimates (dependent variable: Obesity, independent variables: Non-Hispanic Black, non-Hispanic White, Hispanic, median age, bachelor’s degree or higher, female, unemployed, median household income, vehicle ownership, accessible recreational areas, people living in food desert area, fast-food restaurants). tigris [60] package in R was used to download State and County shapefiles and tmap [61] package in R was used to create a figure.

Based on the GWR parameter estimates in Table 6, we mapped local coefficients between independent variables and obesity across the contiguous U.S. We visualized coefficients that are statistically significant at 0.05 level based on absolute value of t-values equal to or greater than 1.96. We mapped local coefficients of park accessibility, food deserts exposure, and density for fast-food restaurants for obesity in Fig 3(A)-3(C).

**Fig 3:** GWR estimates between park access and obesity. **(a).** tigris [60] package in R was used to download State and County shapefiles and tmap [61] package in R was used to create a figure. **(b). GWR estimates between the food deserts exposure and obesity.** tigris [60] package in R was used to download State and County shapefiles and tmap [61] package in R was used to create a figure. **(c). GWR estimates between fast-food restaurants density and obesity.** tigris [60] package in R was used to download State and County shapefiles and tmap [61] package in R was used to create a figure.

**Table 6:** Local coefficient summary (GWR-obesity).

Variables	Min	1st quartile	Median	3rd quartile	Max
% Black	-2.663	-0.465	0.611	1.291	4.455
% Hispanic	-2.892	-0.914	-0.533	-0.335	2.222
% White	-3.283	-0.853	-0.397	-0.307	5.247
Median age	-0.469	-0.280	-0.203	-0.158	0.153
% Bachelor’s degree or higher	-0.941	-0.571	-0.445	-0.341	-0.186
% Female	-0.317	0.116	0.153	0.206	0.362
% Unemployed	-0.427	-0.275	0.136	0.270	0.883
Median household income ($)	-0.413	-0.281	0.166	0.241	0.394
% Vehicle ownership	-0.434	-0.200	0.164	0.250	0.599
% Accessible park areas	-1.300	-0.406	-0.295	-0.205	0.141
% People living in food desert area	-0.320	-0.185	0.106	0.157	0.302
Density of fast-food Restaurants	-0.148	-0.089	0.152	0.190	0.310

Fig 3(A) shows the spatial pattern of GWR estimates between park access (PA) and obesity. Coefficients of park accessibility with a negative direction for obesity (-1.300 to -0.639) are displayed in parts of states including Kansas, Mississippi, Oklahoma, Texas, and large areas in Alabama. Largely, counties with statistically significant coefficients of park access show a negative direction to obesity.

Fig 3(B) illustrates the spatial pattern of GWR estimates between food deserts exposure and obesity. A few counties in states including Alabama, Colorado, Georgia, Kentucky, Pennsylvania, Tennessee, Virginia, and Wyoming present coefficients with positive direction for obesity (0.130 to 0.302). However, some counties in Illinois, Indiana, Kentucky, Michigan, and South Carolina show coefficients with negative direction for obesity (-0.320 to -0.169), indicating that the degree and direction of the association between food deserts exposure and obesity varies significantly across the U.S.

Fig 3(C) depicts local coefficients of the density of fast-food restaurants (FFR) on obesity. High coefficients with positive direction (0.152 to 0.310) are concentrated in parts of Illinois, Kentucky, Missouri, and New York, and in most counties of Pennsylvania. Coefficients with negative direction (-0.148 to -0.094) are in areas that border South Dakota and Wyoming, and parts of California, Nevada, North Carolina, Oklahoma, and Virginia. Like the map of GWR estimates for food deserts exposure and obesity, the spatial pattern of high and low coefficients of the density of FFR for obesity tells the extent and direction of local coefficients differ greatly across the U.S.

Local R-squared values of GWR using diabetes as the independent variable are displayed in Fig 4. Parts of Rocky Mountain states, Midwest states, and Southern states, especially most states that formed the historic cotton belt, present the highest R-squared values (0.754 to 0.844). Counties with the lowest R-squared values (0.447 to 0.598) are clustered in the Appalachian and Midwest states such as Illinois, Indiana, Kansas, Kentucky, Nebraska, Tennessee, and West Virginia.

**Fig 4:** Local R-squared estimates (dependent variable: Diabetes, independent variables: Non-Hispanic Black, non-Hispanic White, Hispanic, median age, bachelor’s degree or higher, female, unemployed, median household income, vehicle ownership, accessible recreational areas, people living in food desert area, fast-food restaurants). tigris [60] package in R was used to download State and County shapefiles and tmap [61] package in R was used to create a figure.

Using the five-number summary of GWR parameter estimates in Table 7, local coefficients between independent variables and diabetes were mapped in Fig 5(A)-5(C). Fig 5(A) shows spatial heterogeneity of the association between PA and diabetes based on the range of local coefficients (-1.164 to 0.170). The lowest GWR estimates (-1.164 to -0.518) are from counties in Alabama, Florida, Kansas, New Mexico, Oklahoma, and Texas. Across the U.S, a greater number of statistically significant local coefficients present a negative direction to obesity.

**Fig 5:** GWR estimates between park access and diabetes. **(a).** tigris [60] package in R was used to download State and County shapefiles and tmap [61] package in R was used to create a figure. **(b). GWR estimates between the food deserts exposure and diabetes.** tigris [60] package in R was used to download State and County shapefiles and tmap [61] package in R was used to create a figure. **(c). GWR estimates between fast-food restaurants density and diabetes.** tigris [60] package in R was used to download State and County shapefiles and tmap [61] package in R was used to create a figure.

**Table 7:** Local coefficient summary (GWR-diabetes).

Variables	Min	1st quartile	Median	3rd quartile	Max
% Black	-3.447	-0.855	-0.293	0.687	1.951
% Hispanic	-2.828	-0.636	-0.455	-0.376	1.353
% White	-3.124	-0.741	-0.491	-0.375	1.111
Median age	0.083	0.209	0.260	0.314	0.579
% Bachelor’s degree or higher	-0.722	-0.430	-0.327	-0.264	-0.139
% Female	0.079	0.115	0.137	0.174	0.328
% Unemployed	-0.641	-0.155	0.159	0.246	0.598
Median household income ($)	-0.520	-0.309	-0.228	-0.179	0.340
% Vehicle ownership	-0.265	-0.166	0.172	0.217	0.311
% Accessible park areas	-1.164	-0.334	-0.191	-0.138	0.170
% People living in food desert area	-0.367	-0.142	0.122	0.219	0.426
Density of fast-food Restaurants	-0.206	-0.089	0.092	0.134	0.273

GWR estimates for the food deserts exposure and diabetes are shown in Fig 5(B). Coefficients with positive direction (0.207 to 0.426) are in counties near the Appalachian region and south Florida. Coefficients with negative direction (-0.367 to -0.177) are in areas that border Illinois, Indiana, and Kentucky. The spatial pattern of high and low coefficients illustrates that the degree and direction of the link between food deserts exposure and obesity varies substantially.

Fig 5(C) illustrates GWR estimates of the density of FFR on diabetes. The highest coefficients with positive direction (0.188 to 0.273) are from a few counties in Illinois, New York, Ohio, and Pennsylvania. Coefficients with negative direction (-0.206 to -0.097) are observed from Mississippi and Oklahoma. The spatial pattern of high and low coefficients and the varying direction of the association between the density of FFR and diabetes confirms the presence of a high degree of spatial heterogeneity.

## 4. Discussion and conclusion

The purpose of this study was to identify spatial clusters of food environment (FE) and park access (PA) that correlate with obesity and diabetes; examine the relationship of the FE and PA with obesity and diabetes from a global regression model; and assess the spatial heterogeneity of environmental variables to diabetes and obesity across the U.S. The result of BiLISA analysis indicates there exists significant spatial variation regarding clusters of environmental variables and dependent variables. This variation is more complex from FE measures than PA measures considering the clustered pattern of each BiLISA cluster. For example, spatial clusters of the FE do show some clustering patterns that we expect such as counties with a high degree of food deserts exposure and the density of fast-food restaurants (FFR) spatially correlating with neighboring counties with high obesity and diabetes rates. LH clusters of the PA measure, however, show relatively more evident spatially clustered patterns. These results imply that PA may be a more important environmental factor than FE in understanding obesity and diabetes.

A global regression model from SEM shows that PA has a statistically significant inverse relationship with obesity and diabetes whereas the FE has a non-significant relationship with both diseases. These findings are consistent with recent studies, which reported non-significant links between obesity and the availability of fast-food restaurants (FFR), grocery stores, and supermarkets [67, 68]. Furthermore, our findings were similar to those studies documenting that diabetes had no significant association with access to supermarkets as well as the density of FFR [69, 70]. Our findings also align with previous studies reporting that obesity and diabetes have a negative relationship with the availability of parks, green space, forest land, and recreation facilities [31, 71–73].

However, as described in a systematic literature review [74], increase in physical activity resources may not lead to reduction in diabetes. We believe these mixed outcomes may occur because the unit of analysis, data included in the research, and the way park accessibility are measured can vary between studies. Our findings will help future systematic literature review or scoping review study when summarizing mixed outcome derived from using different park accessibility measures and food environment exposures.

Although global regression results did not support hypothesis (A) and (B), in which we assumed the FE would show a positive association with obesity and diabetes, at the county level, there exist certain counties that support the hypothesis. The spatially varying relationship between FE and two diseases confirms the importance of incorporating spatial context as it helps locate specific counties where local actions to create more supermarkets and to reduce the unhealthy food outlets would produce promising health outcomes. Among southern states that show high obesity and diabetes rates based on 2019 County Health Rankings data (see Fig 6(A) and 6(B)), Alabama, Georgia, and Kentucky should try eliminating food deserts to reduce the prevalence of obesity and diabetes. Similarly, counties in northwest Pennsylvania, west New York, northeast Ohio, and north Illinois near Chicago may lower diabetes prevalence by reducing the density of FFR. Local coefficients of park access and obesity and diabetes point to areas that need more parks that are accessible. Counties from southern Arizona and southern New Mexico, counties that are connected from Texas to North Dakota, and counties in Alabama and south Mississippi particularly need more accessible parks to lower the risk of developing obesity. Counties in southern New Mexico, counties near west Oklahoma that share a border with Oklahoma and Texas, and counties in Alabama, northwest Florida, and south Mississippi may need more accessible parks to prevent diabetes.

**Fig 6:** Choropleth map of obesity in 2019. **(a).** tigris [60] package in R was used to download State and County shapefiles and tmap [61] package in R was used to create a figure. **(b). Choropleth map of diabetes in 2019.** tigris [60] package in R was used to download State and County shapefiles and tmap [61] package in R was used to create a figure.

The result of the study supports hypothesis (C) and (D) as park access showed inverse relationship with obesity and diabetes from both global and local regression. The findings collectively call for more efforts to promote the access and availability of parks to prevent both diseases. States and municipalities should put more effort into securing funds, such as applying to Outdoor Recreation Legacy Partnership grant authorized by The Land and Water Conservation Fund [75], or developing partnerships with nonprofit organizations (e.g., Trust for Public Land) to increase parks in areas that lack thereof. If developing new parks requires a long-term effort to secure funds and available lands to build, as a short-term approach, opening schoolyards to the community for recreational purposes may help resolve the issue of limited access to the park [76].

Based on choropleth maps of obesity and diabetes shown in Fig 6(A) and 6(B), bivariate LISA clusters, and GWR analysis, high prevalence of both diseases (especially diabetes) in counties of north Alabama is associated with high food deserts exposure and limited park access in those counties. This result aligns with the findings from a recent study [77], which show cities in the southern U.S lack access to health-promoting resources (i.e., supermarkets, recreational green space) and the “multiple-deserted areas” lead to higher prevalence of obesity and diabetes compared to non-multiple-deserted areas. Future studies should use more fine-scale demographic and environmental data to examine which census block groups or tracts in north Alabama are suffering from obesity and diabetes due to compounded disadvantage in access to healthy foods and recreational resources.

GWR estimates for the food deserts exposure showed an inverse relationship with both obesity and diabetes in Illinois, Indiana, and Kentucky. This result is different from the hypothesis we presented. In future studies, obtaining more detailed food environment information (more fine scale than county levels) may help better understand why south Illinois, south Indiana, and northwest Kentucky, that are close to each other show inverse relationship between food deserts exposure and obesity/diabetes.

Although the current study presents some unique findings, it also has several limitations. Regarding FE measures, we did not include other measures such as farmer’s market, convenience stores, and small independent grocery stores. Future studies should incorporate these measures to reflect a more comprehensive FE. If people frequently use these alternative food resources to purchase healthy or unhealthy food, it will help explain the underlying factors that may result in an insignificant association between FE measures we used (percent of people living in food desert area and density of FFR) and obesity and diabetes. Further, this study did not include the price of items in supermarkets, which can be a defining factor of visitation. Future studies should incorporate factors that could affect perceived access to groceries and supermarkets in conjunction with physical access to gain a deeper understanding of supermarket visits. Additionally, this study focused on PA and did not account for more context-specific information about parks and recreation facilities such as their size, quality, operational funding, and crime rates in and around those spaces [78, 79]. As these factors related to the quantity and quality of park could function as a moderator or mediator of the relationship of PA with obesity and diabetes in the U.S, future national-level studies may incorporate these indices in their analysis to discover more clear relationships between PA, diabetes, and obesity.

As diabetes data is self-reported, we acknowledge that data of certain respondents may either overestimate or underestimate the true measures. For example, certain demographic groups can be underrepresented because they are largely absent from home during daytime hours when the survey was conducted. Furthermore, individuals may be unaware of their diabetic status, which can lead to potential inaccuracies in data.

One of the outcome variables, density of fast-food restaurants, is subject to ‘edge effects’ issue that can arise regarding the geographic boundary of unit of analysis. The presence and close accessibility to abundant fast-food restaurants in neighboring counties, particularly near geographic borders, can have an impact on residents living in counties with a comparatively lower density of such restaurants. As we did not address this potential edge effect, we recommend future studies collect fast-food restaurants data from OpenStreetMap as it provides the actual location of individual fast-food restaurants. Studies can address a potential edge effect issue by accounting for the presence of fast-food restaurants in adjacent administrative units.

Lastly, since this study adopts ecological study design, in which the data is aggregated at the geographic level and population level, findings cannot be generalized at individual level. Similarly, due to this study being cross-sectional, our results do not establish causal relationship between variables. Future studies may consider quasi-experimental time series analysis to confirm whether improving park access can reduce obesity and diabetes.

Despite these limitations, this study has several strengths. First, this is the first study that used bivariate LISA, spatial regression, and GWR to explore spatial clusters in the U.S where FE and PA spatially correlate with obesity and diabetes, and analyzed the association between those environmental variables, diabetes, and obesity both in global and local levels. Second, this study confirmed that between food desert exposure, density of fast-food restaurants, and park access, park access plays a more important role in predicting obesity and diabetes at the global level compared to the other measures. Finally, this study contributes to a growing body of research reporting the presence of an obesity and diabetes belt in the U.S South by presenting specific environmental amenities that can lower the risk of developing obesity and diabetes as well as identifying specific states that need those amenities the most. It turns out that improving physical access to parks, particularly in Alabama and Mississippi, might help reduce obesity and diabetes largely than in other states.

We hope that findings from this study help policymakers and public health agencies determine which geographic areas need to be prioritized when implementing public interventions such as promoting healthy food access, limiting unhealthy food options, and increasing park access. We hope our results advocate the necessity of increasing accessible parks to address the issue of health disparities especially in southern U.S.
